The article "Cornuside Alleviates Diabetes Mellitus-Induced Testicular Damage by Modulating the Gut Microbiota" was published in 2021. Journal: Evid Based Complement Alternat Med.

# Cornuside Alleviates Diabetes Mellitus-Induced Testicular Damage by Modulating the Gut Microbiota

**DOI:** 10.1155/2021/5301942

**Published:** 2021-08-30

**Authors:** Liping Liu, Anmei Shu, Yihui Zhu, Yuping Chen

**Affiliations:** ^1^College of Pharmacy, Jiangsu Vocational College of Medicine, #283 Jiefang South Road, Yancheng 224000, Jiangsu, China; ^2^College of Pharmacy, Nanjing University of Chinese Medicine, Nanjing 210023, Jiangsu, China; ^3^Department of Basic Medical Science, Jiangsu Vocational College of Medicine, Yancheng 224005, Jiangsu, China

## Abstract

**Background:**

Male reproductive damage, as a common complication of diabetes mellitus (DM), is getting more attention lately. We aimed to explore the protective effects and mechanism of cornuside (Cor) modulating gut microbiota to alleviate diabetes mellitus- (DM-) induced testicular damage.

**Methods:**

KK-Ay mice with reproductive damage were randomly divided into the model and Cor treatment groups, and the C57BL/6J mice were used as the normal group. These mice were orally administered Cor for 8 weeks.

**Results:**

Cor administration ameliorated the diabetes-related symptoms of polydipsia and polyphagia and lowered the fasting blood glucose (FBG) level. The results of pathological injury showed that Cor improved testicular lesions (the rupture of seminiferous tubules, degeneration of germ cells, and structural shrinkage and separation from each other) in DM model mice. Cor significantly increased the testis/body weight ratio, testosterone, luteinizing hormone (LH), and follicle-stimulating hormone (FSH) levels in KK-Ay mice. Cor also protected from reproductive damage by inhibiting apoptosis in the testes of KK-Ay mice. Moreover, Cor significantly increased the sperm count and sperm motility. Additionally, 16S rDNA sequencing analysis showed that Cor could notably reverse the changes in the distribution of gut microbiota and decrease the abundance of *Weissella confusa* (*Weissella*), *Clostridium* sp. ND2 (*Clostridium* sensu stricto 1), uncultured bacterium *(Roseburia*), *Anaerotruncus colihominis* DSM 17241 (*Anaerotruncus*), [*Clostridium*] *leptum* (*Anaerotruncus*), unidentified (*Ruminococcus* 1), and uncultured bacterium (*Bilophila*), which may be a potential biomarker for diagnosing the testicular injury caused by DM. Meanwhile, the heat map of phylum level suggested that the testicular injury caused by DM is closely related to gut microbiota.

**Conclusions:**

Cor could alleviate DM-induced testicular damage, probably by modulating the gut microbiota.

## 1. Introduction

Diabetes mellitus (DM) is a common metabolic disease affecting more than 451 million adults aged >18 years as of 2017, and this number is projected to rise to 693 million by 2045 [1]. The change in people's lifestyle and the trend of population aging with the economic development have led to an increase in the incidence of DM every year. Increasing attention has been paid to the DM-induced reproductive injury besides the well-known damage to the cardiovascular and renal systems. Accumulating evidence suggests that humans and diabetic experimental animals with DM have changes in reproductive function, particularly in spermatogenesis, testicular histology, steroidogenesis, sperm quality, and fertility [2–6]. DM accompanied by persistent hyperglycemia can cause testicular damage by causing erectile dysfunction, retrograde ejaculation, and loss of libido, leading to male infertility [7–9]. DM is a vital factor for male infertility; however, the underlying mechanism remains unknown.

Gut bacteria participate in metabolism, including the regulation of intestinal motility, synthesis of micronutrients, and fermentation of undigested carbohydrates, thereby playing a significant regulatory role in DM [10]. The disturbance in the “beneficial” gut microbiota may accelerate the development of DM [11]. The “gut-brain axis” has demonstrated that the intestinal flora influences brain function and activity [12–14], and the hypothalamus-pituitary-testis (HPT) axis is considered to be a classic neuromodulation pathway in steroid production. Therefore, the gut microbiota-testis axis may participate in DM-induced reproductive damage [15]. However, whether DM can cause reproductive damage through gut microbiota is still unknown. Therefore, modulating the gut microbiota may be considered to be an effective treatment for DM-induced reproductive damage.

Modern pharmacological research shows that the Chinese Herbal Medicine *Cornus officinalis* Sieb. et Zucc (CO) and its active ingredients have cardioprotective, antioxidant, anti-inflammatory, anti-aging, neuroprotective, and antibacterial effects to treat DM and other diseases [16]. Besides treating DM-induced reproductive dysfunction using Chinese Herbal Medicine formula (Liu Wei Di Huang Wan pills) [17], an accumulating body of evidence has shown the use of CO for treating patients with DM. Recent studies reported that Liu Wei Di Huang Wan decoction and its active ingredients ameliorated cognitive deterioration via gut microbiome [18, 19].

CO is an important component of Liu Wei Di Huang Wan decoction. Few studies reported that CO could regulate diseases by improving gut microbiota. However, the CO extract could reduce DM-induced testis injury [20, 21]. Cor is one of the effective ingredients extracted from the Chinese Herbal Medicine CO. It has immunomodulatory and anti-inflammatory activities [22, 23]. However, whether Cor has a protective effect on DM-induced testicular damage by modulating the gut microbiota is still unknown. In this study, KK-Ay mice were used to explore the function and mechanism of Cor modulating gut microbiota to alleviate DM-induced testicular damage. The findings might provide new treatments for the use of Cor to treat DM-induced male infertility.

## 2. Materials and Methods

### 2.1. Materials

Cornuside (Figure 1(a); HPLC ≥98% purity) was obtained from Chengdu Ruifensi Biotechnology Co. Ltd. (Chengdu, China). The hematoxylin and eosin (H&E) assay kit was purchased from Beijing Solarbio Science & Technology Co. Ltd. (Beijing, China). The testosterone ELISA kit was obtained from Anhui Joyee Biotechnics Co. Ltd. (Hefei, China). Luteinizing hormone (LH) and follicle-stimulating hormone (FSH) ELISA kits were obtained from Shanghai Meilian Biotechnology Co. Ltd. (Shanghai, China). The TUNEL assay kit was obtained from Beyotime Biotechnology Co. Ltd. (Shanghai, China).

### 2.2. Animal Experimental Procedures

In this study, 14-week-old male KK-Ay and C57BL/6J mice were purchased from Beijing Huafukang Bioscience Co. Ltd. (Beijing, China) (license no. SCXK Beijing 2014-0004). They were housed in a standard animal care facility (25°C ± 1°C; 55% ± 5% relative humidity; and 12-h light/dark cycle). The flow diagram of the animal experiment design is demonstrated in Figure 1(b). The animals were given a 2-week acclimatization period prior to experimental use. The Animal Ethics Committee of the Nanjing University of Chinese Medicine approved the present study (approval number: ACU-13 (20161011)).

According to a random grouping number table, KK-Ay mice were randomized into two treatment groups (*n* = 6/group): the model (DM) group and the cornuside treatment (Cor) group, both fed daily a high-fat diet. The Cor group received cornuside [100 mg/(kg day)] by oral administration, and the DM group received the same volume of normal saline daily equal to that of the Cor group. Six C57BL/6J mice were used as the normal group, which were fed with a normal diet and given the same volume of normal saline daily equal to that of the other groups for an 8-week period. During this period, a high-fat diet (60.5% standard rat feed, 10% sugar, 0.2% cholesterol, 24% lard, and 5% egg yolk powder) obtained from Beijing Huafukang Bioscience Co. Ltd. (Beijing, China) was fed to KK-Ay mice, whereas C57BL/6J mice were fed standard chow. The fasting plasma glucose level in all animals was measured after 4 and 8 weeks using blood collected from the tail vein of these animals following a 12-h fasting period. In addition, the bodyweight, 24-h food consumption, and 24-h water intake were measured. Prior to the sacrifice, the fecal sample of each mouse was collected and stored at −80°C for the analysis of gut microbiota. Also, testis and epididymis were collected and tested.

### 2.3. Histopathological Evaluation

After fixation using 10% formalin, the testicular tissue sections were paraffin-embedded, cut into 5 *μ*m sections, and stained using H&E. A microscope was then used to evaluate islet histology (200×). Images were blindly taken from randomly selected areas, and the representative images of these parts were displayed. Testicular tissue injury was analyzed and semiquantitatively scored by pathologists on the basis of the hierarchical arrangement and structure of spermatogenic cells, interstitial vasodilation, interstitial cell hyperplasia, hemorrhage, and inflammatory cell invasion. Data were presented as mean ± SEM. A score of 0 represented no lesions, and a score of 6 represented the most severe lesions.

### 2.4. Measurement of Testosterone, LH, and FSH Levels

The testosterone, LH, and FSH levels in testes were assessed following the manufacturer's protocols. In brief, the samples were added for 2 h at 28°C to 96-well plates coated with primary antibodies. Then, the wells were washed three times, and a 100 *μ*L volume of the chromogenic substrate was added for 20 min at 28°C. The absorbance at 450 nm was then evaluated within 10 min of the addition of 50 *μ*L of stop solution to each well.

### 2.5. Measurement of the Apoptosis of Testicular Cells in KK-Ay Mice

The TUNEL assay was used for testing apoptotic testicular cells. After fixation using 10% paraformaldehyde, the testicular tissue sections were paraffin-embedded and cut into 5 *μ*m sections. In brief, the testicular tissue sections were dewaxed, rehydrated in xylene and ethanol, and then incubated with the working solution of proteinase K at 37°C for 20 min. Further, 50 *μ*L of TUNEL reaction mixture was added after washing the samples with PBS at 37°C for 1 h. The samples were again washed with PBS to stop the reaction. Apoptosis was found to occur in TUNEL-positive cells. ImageJ software was used for quantitative analysis.

### 2.6. Measurement of Sperm Count and Sperm Motility

The epididymis was cut, and the sperm suspension was dissolved in saline. The sperm suspension was placed in the Neubauer counting chamber, and the sperms were counted by using a light microscope. Sperm motility was detected by eosin-nigrosin one-step staining technique and distinguished by staining (Bjorndahl et al. 2003).

### 2.7. Extraction of Fecal Genomic DNA and Sequencing

Fecal DNA was extracted from cecum stool samples using E.Z.N.A. soil kit (Omega Bio-Tek, GA, USA) following the manufacturer's instructions. The hypervariable V3-V4 region of the 16S-rDNA gene was amplified by PCR using the primers 338F: 5′-ACTCCTACGGGAGGCAGCAG-3′. The cycling conditions were as follows: initial denaturation at 95°C for 3 min, 28 cycles of denaturation at 95°C for 30 s, annealing at 55°C for 30 s, elongation at 72°C for 45 s, and final extension at 72°C for 5 min and 10°C until completion. Amplicons were recovered from 2% agarose gels and purified using an AxyPrep DNA Gel Extraction Kit (Axygen Biosciences, CA, USA) following the manufacturer's instructions and quantified using a QuantiFluor-ST fluorometer (Promega, USA). The purified amplicons were pooled in equimolar ratio and paired-end sequenced (2 × 300 bp) using PE300 strategies on an Illumina MiSeq platform (Illumina, CA, USA). The raw reads were deposited into the NCBI Sequence Read Archive database (accession number: SRP168312).

### 2.8. Bioinformatics Analysis

Illumina paired-end reads were connected, filtered, and then processed using the software package of QuantiFluor-ST. Sequences with ≥97% similarity were assigned to the same operational taxonomic units (OTUs). The representative sequences for each OTU were screened, and the differential analysis of groups of dominant species was performed. Alpha and beta diversities were used to analyze the complexity of species diversity.

### 2.9. Statistical Analysis

Data were expressed as mean ± SD and compared using one-way ANOVA with Tukey's post hoc test. SPSS 22.0 was used for all statistical analyses, and *P* < 0.05 indicated a statistically significant difference. SPSS was used to calculate Pearson's correlation coefficient to verify the correlation between bacterial abundance and reproductive injury indexes such as FBG, testicular index, testosterone, and live sperm rate. GraphPad software was used to draw a heat map of Pearson's correlation coefficient between the above indexes and bacterial abundance.

## 3. Results

### 3.1. Cor Improved General Symptoms of KK-Ay Mice

The 24-h food consumption, 24-h water intake, FBG, and body weight were measured in all experimental animals after 0, 4, and 8 weeks of the study. The 24-h food consumption and 24-h water intake dramatically increased in the DM model mice compared with the control mice in the 8th week (Figures 1(c) and 1(d)). Moreover, the FBG level remarkably improved in the model group compared with the control group, which was markedly decreased by Cor treatment (Figure 1(e)). Cor administration ameliorated the symptoms of polydipsia and polyphagia and increased the body weight compared with those in the DM model mice (Figure 1(f)).

### 3.2. Cor Mitigated Testicular Lesions in KK-Ay Mice

The study next analyzed testicular tissue and testis/body weight ratio. H&E staining was used to assess morphological changes so as to examine how Cor treatment affected testicular histopathology in DM model mice. The testis of mice in the control group showed normal testicular tissue structure, including concentric layers of integral seminiferous tubules and organized germ cells. Spermatogenic cells in various stages, spermatogonia to spermatids, were observed, accompanied by some interstitial cells in the lumen of neatly arranged seminiferous tubules. The mice in the DM model group exhibited rupture of seminiferous tubules, degeneration of germ cells, and structural shrinkage and separation from each other. The pathological injury was remitted to different degrees after an 8-week treatment with Cor.  Figure 2(a) shows the pathological score of testicular lesions. Additionally, the testis/body weight ratio significantly decreased in the DM model group compared with the control group (Figure 2(b)), while it significantly increased in the Cor group compared with the DM model mice. Testosterone is crucial in sperm production, formation, and maturation. It is mainly secreted by testicular interstitial Leydig cells and closely related to spermatogenesis (Wang et al. 2009). The testosterone level represents sperm motility to some extent. The testosterone level in testes among groups is shown in Figure 2(c). The testosterone level significantly decreased in the DM model group compared with the control group, which was significantly increased by Cor treatment. Consistent with the testosterone trend, the LH and FSH levels also significantly decreased in the DM model group compared with the control group, which was significantly increased by Cor treatment (Figures 2(d) and 2(e)).

### 3.3. Cor Ameliorated the Apoptosis of Testicular Cells in KK-Ay Mice

TUNEL assay was used to assess apoptosis so as to examine the anti-apoptotic effect of Cor treatment on testicular injury in KK-Ay mice. The DM model mice exhibited a large number of apoptotic cells in the testes compared with normal mice; the apoptosis was mitigated by Cor administration (Figures 3(a) and 3(b)). Therefore, Cor had anti-apoptotic effects on DM-induced testicular damage.

### 3.4. Cor Improved the Sperm Count and Sperm Motility

Sperm count and sperm motility were tested after the experiment; the sperm count and sperm motility were significantly reduced in the DM model group compared with the control group, which was significantly increased by Cor treatment (Figures 3(c) and 3(d)).

### 3.5. Cor Improved the Dysbiosis of Gut Microbiota in KK-Ay Mice

16S rDNA sequencing analysis was performed to detect the changing characteristics of gut microbiota so as to investigate the influence of DM-induced intestinal flora dysbiosis on testicular damage. The OTU clustering of unique sequences was based on 97% sequence similarity. Alpha diversity of the gut microbiota was determined using the Chao index, Shannon index, and rarefaction curve. The alpha diversity dramatically reduced in the DM model group compared with the control group (*P* < 0.05). At the same time, Cor treatment could notably restore the alpha diversity of DM model mice. The dynamics of alpha diversity indices, including Chao index and Shannon index, indicated that the abundance and diversity of gut bacteria increased significantly in the Cor group compared with the DM model group (Figures 4(a) and 4(b)). Moreover, the number of OTUs observed was lower in the model group than in the other two groups. The rarefaction curve analysis showed that the sequencing depth covered rare new phenotypes and species as far as possible (Figure 4(c)). As shown in Figure 4(d), a weighted PCoA clearly demonstrated the compositional differences in gut microbiota with an obvious difference along the PC1 axis (reaching 49.4% of overall variation).

The results of the hierarchical cluster tree analysis showed significant clustering between the control and model groups; the Cor group also showed a better separation trend (Figure 5(a)). LEfSe was used to identify the bacterial phenotypes with specific changes from phylum to genus so as to study further the differences among control, model, and Cor groups. The cladogram showed the dominant bacteria in each group (Figure 5(b)). The LDA score (log 10 > 2) showed significant changes in 68 bacteria in the 3 groups (Figure 5(c)). The composition of gut bacterial species in each group showed apparent differences. Differential microbial lineages in the control group included 20 bacteria belonging to *Verrucomicrobiales*, *Akkermansia*, *Verrucomicrobia*, *Verrucomicrobiaceae*, *Verrucomicrobiae*, *Actinobacteria*, *Bifidobacteriaceae*, and so forth. Differential microbial lineages in the model group included 30 bacteria belonging to *Enterobacteriales*, *Gammaproteobacteria*, *Enterobacteriaceae*, Escherichia Shigella, *Enterococcaceae*, *Enterococcus*, and so forth. Differential microbial lineages in the Cor group included 18 bacteria belonging to *Rikenellaceae*, *Alistipes*, *Ruminiclostridium*_5, *Lachnospiraceae*_UCG_001, *Butyricicoccus*, *Odoribacter*, *Marvinbryantia*, and so forth.

### 3.6. Cor Reverses the Changes in the Distribution of the Microbes in KK-Ay Mice

It is worth noting that among the 68 strains of microorganisms, 7 strains are significantly different among the 3 groups, including *Weissella confusa* (*Weissella*), *Clostridium* sp. ND2 (*Clostridium* sensu stricto 1), uncultured bacterium (*Roseburia*), *Anaerotruncus colihominis* DSM 17241 (*Anaerotruncus*), [*Clostridium*] *leptum* (*Anaerotruncus*), unidentified (*Ruminococcus* 1), and uncultured bacterium (*Bilophila*) (Figures 6(a)–6(g)). Interestingly, the relative abundance of the marked 7 strains of microorganisms were significantly increased, which were significantly decreased by Cor treatment. These results suggest that Cor reverses the changes in the distribution of these microbes, which may be a potential biomarker for diagnosing the testicular injury caused by DM.

### 3.7. Correlation Analysis of Different Flora and Reproductive Injury Indexes

In order to explore the relationship between the testicular injury caused by DM and gut microbiota, we analyzed the correlation between gut microbiota, FBG, testicular index, testosterone, and live sperm rate. As shown in Figure 7(a), the closer the color is to red, the greater the positive correlation between the two parameters, and the closer the color is to blue, the greater the negative correlation between the two parameters in the heat map. The heat map suggested that *Akkermansia*, *Bacteroidales* S24-7 group, and *Lachnospiraceae* were negatively correlated with FBG. *Akkermansia*, *Bacteroidales* S24-7 group, *Lactobacillus*, *Bacteroidaceae*, and *Prevotellaceae* were positively correlated with testicular index, while *Roseburia* were negatively correlated with testicular index. *Alloprevotella* was positively correlated with testosterone, while *Roseburia* were negatively correlated with testosterone. *Bacteroidales* S24-7 group, *Akkermansia*, and *Bacteroidaceae* were positively correlated with live sperm rate, while *Prevotellaceae* were negatively correlated with live sperm rate.

As shown in Figure 7(b), the heat map of phylum level suggested that *Bacteroidetes* were positively correlated with FBG. *Bacteroidetes* were negatively correlated with testicular index. *Actinobacteria* were positively correlated with testosterone. *Bacteroidetes* were negatively correlated with live sperm rate, while *Firmicutes* were positively correlated with live sperm rate. These results suggest that the testicular injury caused by DM is closely related to gut microbiota.

## 4. Discussion

DM, as a common metabolic disease, causes numerous organ and system dysfunctions, including the male reproductive system [24]. Gut microbiota are believed to be vital in regulating DM [25]. They also affect other systems, such as the nervous system and reproductive system [26, 27]. They affect the reproductive performance in men and women [28]. The present study investigated whether DM-induced intestinal flora alteration was one of the important causes of the reproductive damage. The findings established a functional linkage between gut microbiota dysbiosis and DM-induced male reproductive injury. Moreover, this study proved the therapeutic effect of Cor on DM-induced male reproductive damage, and this reproductive protection was closely related to the modulation of gut microbiota.

In this study, a KK-Ay spontaneous DM mouse model system was used to evaluate the impact of Cor on disease progression. These mice were selected because they exhibit traits consistent with type 2 DM in humans. The study showed typical symptoms of DM, including polydipsia, polyphagia, weight loss, and elevated FBG levels, along with morphological and functional impairment of the reproductive system, in male KK-Ay mice. The effect of the gut microbiome on diseases has gained interest with the development of modern medicine. Recent studies showed that the abundance of *Bacteroides* and *Prevotella* strongly negatively correlated with sperm motility while the abundance of *Bacteroides* strongly positively correlated with the blood endotoxin concentration in male infertile patients with asthenozoospermia/oligozoospermia/teratozoospermia [29]. Interestingly, we also found that *Bacteroidetes* were also strongly negatively correlated with testicular index and live sperm rate. The gut microbiota-testis axis may modulate DM-induced reproductive damage according to the concept of the gut-brain axis and the HPT axis. The present study found that the testicular tissue of the DM model mice exhibited the rupture of seminiferous tubules, degeneration of germ cells, and structural shrinkage and separation from each other. Meanwhile, the testis/body weight ratio, testosterone, LH, and FSH levels were remarkably lower. Moreover, the DM model mice exhibited a large number of apoptotic cells in the testes. These results indicated obvious male reproductive damage in KK-Ay mice. The results of fecal 16S rDNA gene sequencing analysis showed that the mice with DM-induced reproductive damage had abnormal microbial changes. Both Chao and Shannon indexes showed that the diversity and abundance of gut microbiota were significantly reduced in the model group, and Cor reversed these changes. Interestingly, the relative abundance of the marked 7 strains of microorganisms such as *Weissella confusa*, *Clostridium* sp. ND2, *Anaerotruncus colihominis* DSM 17241, *Clostridium leptum*, and so on were significantly increased, which were significantly decreased by Cor treatment. These results suggest that Cor reverses the changes in the distribution of these microbes, which may be a potential biomarker for diagnosing the testicular injury caused by DM. Sartonoa et al. reported that bacteriocin peptides from *Weissella confusa* MBF8-1 exhibited spermicidal activity by affecting the motility of spermatozoa and sperm [30]. In our study, DM mice exhibited significantly increased abundance of *Weissella confusa* at the species level in DM mice, which might be closely related to the reproductive damage in accordance with Sartonoa's reports. Moreover, the heat map of phylum level suggested that the testicular injury caused by DM is closely related to gut microbiota.

Cor is an active ingredient extracted from the Chinese Herbal Medicine CO. It has immunomodulatory and anti-inflammatory activities. For example, Cor inhibited the expression of pro-inflammatory and adhesion molecules induced by human vascular endothelial cells and protected cultured rat cortical cells [22, 23]. Moreover, it inhibited the production of nitric oxide by lipopolysaccharides in cultured mouse macrophages, thus inhibiting the damage caused by oxygen-glucose deprivation [31]. The CO extract could reduce DM-induced testis injury [20]. Cor is one of the primary bioactive monomers extracted from CO iridoid glycoside, which may also target the testes to improve DM-induced reproductive damage. Moreover, the CO extract, including iridoid glycosides, alcohol extracts, saponins, and tannins, significantly improved the gut microbes in DM mice [32].

The present study found that Cor improved the general diabetes-related symptoms of polydipsia and polyphagia and also the elevation of FBG level in KK-Ay DM mice. Cor also reduced the reproductive damage and histopathological changes in these mice, as proved by testicular lesions, testis/body weight ratio, and tissue apoptosis. Moreover, Cor significantly reversed the flora disorder in mice with DM-induced reproductive damage. The exact mechanism underlying the correlation between testicular damage and gut microbiota is needed to be investigated systematically to clarify that Cor alleviates DM-induced reproductive damage. The present study demonstrated that Cor remarkably improved DM-induced reproductive damage by relieving diabetes-related symptoms, protecting the testicular structure, and reducing testicular cell apoptosis. Cor also significantly reduced the abundance of *Weissella confusa* (*Weissella*), *Clostridium* sp. ND2 (*Clostridium* sensu stricto 1), uncultured bacterium (*Roseburia*), *Anaerotruncus colihominis* DSM 17241 (*Anaerotruncus*), [*Clostridium*] *leptum* (*Anaerotruncus*), unidentified (*Ruminococcus* 1), and uncultured bacterium (*Bilophila*) in the DM model mice. Moreover, the heat map of phylum level suggested that *Bacteroidetes* were positively correlated with FBG. *Bacteroidetes* were negatively correlated with testicular index. *Actinobacteria* were positively correlated with testosterone. *Bacteroidetes* were negatively correlated with live sperm rate, while *Firmicutes* were positively correlated live sperm rate. The results suggested that Cor alleviated DM-induced testicular damage via modulating gut microbiota. However, the mechanism underlying the effect of Cor on DM-induced male reproductive damage needs further exploration.

## Figures and Tables

**Figure 1:** Cor improved the general symptoms in KK-Ay mice. (a) Chemical structural formula of Cor. (b) Flow diagram of animal experiment design. (c) 24-h food consumption. (d) 24-h water intake. (e) Fasting blood glucose level. (f) Body weight; *n* = 6/group; ^*∗∗*^*P* < 0.01 versus the control group; ^##^*P* < 0.01 versus the model group.

**Figure 2:** Cor mitigated testicular lesions and function in KK-Ay mice. (a) (A)–(C) H&E staining images of testicular tissues in each group (200× magnification). (D) Testicular lesion score chart. (b) Cor improved the testis/body weight ratio. (c) Cor elevated the testosterone level in KK-Ay mice. (d) Cor elevated the LH level in KK-Ay mice. (e) Cor elevated the FSH level in KK-Ay mice. ^*∗∗*^*P* < 0.01 versus the control group; ^##^*P* < 0.01 versus the model group.

**Figure 3:** Cor ameliorated testicular cell apoptosis and function in KK-Ay mice. (a) TUNEL staining images of positive cells are displayed in green (white arrow) (200× magnification). Hoechst staining was performed on the cell nuclei. (b) Percentage of apoptotic cells. (c) Cor improved the sperm count of KK-Ay mice. (d) Cor improved the sperm motility of KK-Ay mice. ^*∗∗*^*P* < 0.01 versus the control group; ^##^*P* < 0.01 versus the model group.

**Figure 4:** Cor increased the diversity of the gut microbiota in KK-Ay mice. (a) Chao index chart. (b) Shannon index chart. (c) Rarefaction curve. (d) PCoA plot of each group was generated using operational taxonomic unit metrics based on the Bray–Curtis dissimilarity. The center coordinates of the ellipse are the average values of PC1 and PC2. The values of PC1 and PC2 are displayed in a scatter chart. ^*∗∗*^*P* < 0.01 versus the control group; ^##^*P* < 0.01 versus the model group.

**Figure 5:** Taxonomic differences in gut microbiota among the control, model, and Cor groups. (a) Hierarchical cluster tree. (b) Taxonomic cladogram acquired using LEfSe. Differences are reflected in the color of the richest class (green represents the control group, red represents the model group, and blue represents the Cor group). The diameter of each circle is proportional to the abundance of the taxon. (c) Statistical LDA score (log 10 >2) of significantly acting microbial taxa in different groups obtained using LDA analysis. The ordinate indicates the taxa with significant differences, and the abscissa indicates the LDA scores in the bar graph. The bars are sorted by the score to describe the differences in each sample. The longer the bar, the more significant the difference. ^*∗∗*^*P* < 0.01 versus the control group; ^##^*P* < 0.01 versus the model group.

**Figure 6:** Effect of cor on the relative abundance of different bacteria. (a) Weissella; s Weissellaconfusa. (b) uncultured; s uncultured bacterium. (c) Clostridium sensu stricto 1; s Clostridium sp. ND2. (d) Roseburia; s uncultured bacterium. (e) Anaerotruncus; s Anaerotruncus colihominis DSM 17241. (f) Anaerotruncus; s [Clostridium] leptum. (g) Ruminococcus 1; s unidentified. (h) Bilophila; s uncultured bacterium. ^*∗∗*^*P* < 0.01, ^*∗*^*P* < 0.05 versus the control group; ^##^*P* < 0.01, ^#^*P* < 0.05 versus the model group.

**Figure 7:** Correlation analysis of reproductive injury indexes induced by KK-Ay mice and gut microbiota. (a) Heat map of the correlation between changes in gut microbiota and changes in FBG, testicular index, testosterone, and live sperm rate at OTU level. (b) Heat map of the correlation between changes in gut microbiota and changes in FBG, testicular index, testosterone, and live sperm rate at genus level. ^*∗∗*^*P* < 0.01, ^*∗*^*P* < 0.05 versus the control group; ^##^*P* < 0.01, ^#^*P* < 0.05 versus the model group.

## Data Availability

The data used to support the findings of this study are available from the corresponding author upon request.
